# Dynamic Allocation Method of Economic Information Integrated Data Based on Deep Learning Algorithm

**DOI:** 10.1155/2022/5494123

**Published:** 2022-05-16

**Authors:** Zhitao Cao

**Affiliations:** Baotou Teachers College, Baotou 014030, China

## Abstract

In view of the low efficiency of traditional data fusion algorithms in wireless sensor networks and the difficulty in processing high-dimensional data, a new algorithm CNNMDA, based on the deep learning model is proposed to realize data fusion. Firstly, the algorithm trains the constructed feature extraction model CNNM at the sink node; then each terminal node extracts the original data features through CNNM and finally sends the fused data to the sink node, so as to reduce the data transmission amount and prolong the network life. Simulation experiments show that compared with similar fusion algorithms, the CNNMDA can greatly reduce network energy consumption under the same data amount, and effectively improve the efficiency and accuracy of data fusion. In order to solve the problem that parameter synchronization takes too long in synchronous parallel, a dynamic training data allocation algorithm in multimachine synchronous parallel is proposed. Based on the computing efficiency of compute nodes, the amount of sample data to be processed by nodes will be dynamically adjusted after each iteration. This mechanism not only enables the model to be synchronized and parallel but also reduces the time of waiting for gradient updates. Finally, a comparative experiment is carried out on the Tianhe-2 supercomputer, and the experimental results show that the proposed optimization mechanism achieves the expected effect.

## 1. Introduction

A distributed system consists of a set of compute nodes that communicate and coordinate work across a network to accomplish a common task. The emergence of the distributed system is to use multiple ordinary machines to complete computing and storage tasks that cannot be completed by a single computer. The purpose is to use more machines to process more data. The characteristics of the distributed system fully meet the needs of deep learning. Through the in-depth study on large-scale distributed platforms, we can make full use of distributed hardware and system advantages. On the premise of ensuring the accuracy of training, improving the speed of model training becomes the main goal of distributed deep learning, which is also one of the focuses of this paper.

In this paper, the deep learning framework MXNET, based on the neural network is adopted. Its main advantages are fast training speed and good performance optimization, and it is one of the fastest learning frames of the current machine. Meanwhile, MXNET is based on the architecture of the parameter server, and it also has perfect support for distributed parallel training. The traditional parallel training process of parameter servers can be divided into two modes: synchronous mode and different step mode. The synchronization mode is to update parameters in the form of average aggregation. This method has great limitations, that is, it needs to wait for all computing nodes to train the next batch after training the current batch. Therefore, when the computing speeds of different computing nodes in the cluster are inconsistent, it will cause very serious idle resources and waste of time. In essence, the emergence of asynchronous mode is to solve the above problems. When the gradient update of a computing node is collected, the asynchronous mode updates the parameter once and no longer waits for the rest of the nodes to complete the calculation, which improves the utilization of computing resources. However, the convergence of the model is poor because of the out-of-date gradient generated by some nodes in the asynchronous mode. According to the above problem, this paper presents a dynamic allocation algorithm of multimotor synchronous parallel data, the main design idea is under the data-parallel synchronous mode as far as the shortboard effect, through the data distribution of MXNet module into the line change, the proportion of data distribution from the original average distribution improvement of dynamic allocation. Furthermore, the training time of each node in a single iteration is similar, which greatly improves the training efficiency of the model.

With the rapid development of Internet of Things technology, Wireless Sensor Networks (WSNs), as the core component of the sensing layer of the Internet of Things, has been widely used in various environmental monitoring fields [1]. In practice, most sensor nodes use battery power, which leads to limited resources in the network. Due to the uneven geographical distribution of a large number of nodes, the data have too much redundant information [2], which increase the energy consumption and transmission delay. In addition, due to the widespread interference in the application environment of the Internet of Things, the data communication transmission capacity will be directly weakened, and the accuracy of data acquisition will be reduced, affecting the overall performance of the Internet of Things system. To solve the above problems, the data fusion technology for WSNs emerged. The main idea of the technology is to fuse data from multiple different source nodes to eliminate redundancy and reduce data transmission, so as to improve network performance, extend network life and reduce energy consumption.

Traditional fusion algorithms are mostly based on the BP neural network [3–7], SOFM [8], and other shallow network models, which are prone to overfitting, model training falling into a local minimum, convergence speed is too slow, and other problems, resulting in reduced algorithm efficiency, weak feature extraction, and classification ability, and inability to effectively deal with high-dimensional data. In view of the above defects, the application of the deep model has become a new direction of data fusion development. In 2006, Pinto et al. [9] proposed the concept of “deep learning,” Since then, convolutional neural network (CNN) [10], stack auto-encoder (SAE), and other models have been widely applied. At present, deep learning has been studied in the field of data fusion. References [11] and [12] proposed to use of the SAE model in deep learning to carry out feature fusion of WSNs data, which significantly improved the accuracy of fusion. In literature [13], combined with a deep model and sparse filtering algorithm, the BSSFM model is designed to extract data features, which improves the efficiency of fusion and reduces energy consumption. However, the use of SAE and other models will generate a large number of weight parameters in the training process, which increases the difficulty of model training.

In this paper, the convolutional neural network structure in deep learning is introduced into WSNs' data fusion application. A data fusion algorithm, CNNMDA (convolutional neural network model data aggregation), is proposed, which takes CNNM as the feature extraction model. The algorithm uses the feature of CNN weight sharing to reduce the training parameters, which makes the model easy to train and can better deal with high-dimensional data.

## 2. Dynamic Data Allocation Algorithm Based on Synchronous Parallel Mechanism

The default data allocation mechanism of MXNet is the average data allocation among each node, but the dynamic data allocation algorithm proposed in this paper converts the average data allocation into dynamic data allocation under the synchronization and parallel of multiple machines, so as to improve the efficiency of training.

### 2.1. Processing Process

The main process of the algorithm can be divided into two parts: the computing node side and the parameter server side. This section describes the execution process of the algorithm from the two parts, respectively, and the meanings of relevant parameters involved in the algorithm are shown in Table 1.

The main task of the computing node is to load data at the beginning of the training and initialize the weight of the neural network. In the iteration process, the gradient update and calculation rate are calculated by the forward propagation and backward propagation of the logarithmic data set, which are sent to the parameter server for aggregation and wait for the new model parameters and the new speed direction of the whole office speed rate. Dynamic data adjustment is performed after the end of an epoch. See Figure 1 for the specific process.

The main task of the parameter server node is to aggregate the gradient updates pushed to ensure the consistency of the parameters of the deep neural network on different computing nodes and maintain a global speed vector speed. The specific process within an epoch is shown in Figures 2 and 3.

### 2.2. Research Progress of Deep Learning

Deep learning convolutional neural network (CNN) has been widely used in time series data prediction [3], image processing, and other fields. Applying CNN to financial time series data prediction has the following advantages: firstly, the main advantage of the CNN is that the convolution layer and the pooling layer are used as feature extractors of the input vector, which can learn the important features required for neural network training without providing complex information processing [5]. Secondly, CNN can fully consider the local correlation of temporal or spatial data.

However, it is difficult for CNN to capture the long term sequence characteristics of financial time series data. Scholars have proposed to combine CNN and recurrent neural network incorporating time series data dependence features and apply them to text classification. The cyclic structure captures the context information of words, and CNN automatically determines, which words play key roles in text classification. The verification results show that the classification accuracy of this method is higher than that of a single CNN [6]. Cyclic convolutional neural network can simultaneously process the sequence dependence feature and local association feature of sequence data, and their performance in processing time series data such as text is better than that of existing convolutional neural network. However, whether a cyclic convolutional neural network is applicable to the prediction of financial time series data, and how its prediction effect is compared with the cyclic neural network, have not been explored in the existing literature. Therefore, this paper proposes to combine the CNN with a more simple and effective gated cyclic unit (GRU) neural network of the recurrent neural network, namely, using the CNN_GRU neural network to predict financial time series data [14].

In addition, in the short, medium, and long term, the factors that affect the change of financial time series data are complex and different. In order to improve the prediction accuracy, scholars proposed the combined prediction method of financial time series data by using wavelet analysis, empirical mode decomposition (E Viii), integrated empirical mode decomposition (EEMD), and other methods [7]. EMD and wavelet analysis methods can decompose the information of different frequencies and different amplitudes in the original time sequence data one by one, but the selection of wavelet basis and the selection of decomposition layers will have a great influence on the decomposition results. The decomposition results are not as accurate as the EMD method [8] EEMD can extract the components and variation trends of the time sequence data in an adaptive way, effectively reduce the modal mixing phenomenon in EMD, and overcome the harmonic defects that are easy to occur in wavelet analysis with no physical meaning [9].

Based on the above analysis, the prediction of financial time series data are carried out in this paper from the following two perspectives: First, the CNN-GRU neural network is constructed to analyze the theoretical basis of its application in the prediction of financial time series data. Second, the EEMD and run-length determination methods are used to decompose and reconstruct financial time sequence data into low-frequency components, high-frequency components, and trend terms. Then, machine learning algorithms such as the BP neural network, support vector machine, and deep learning algorithms such as the GRU neural network and the CNN-GRU neural network are used to predict components with different frequencies. Finally, the prediction results of each component are integrated to get the final predicted value of the financial time series data.

## 3. Deep Learning Algorithm Model

Deep learning, a branch of machine learning, has made breakthroughs in many fields in recent years. The convolutional neural network is one of the most important structural models in deep learning.

### 3.1. CNN Concept and Network Structure

Convolutional neural network (CNN) is a multilayer artificial neural network [10]. Its basic network structure includes the convolution layer and the pooling layer. Among them, the convolution layer uses multiple convolution kernels to extract features from the input layer and obtain multiple feature maps. A pooling layer is used to reduce the dimension of the feature map by pooling function, and to control the overfitting as far as possible under the condition of maintaining accuracy, while reducing the number of parameters. The typical structure of convolutional neural network is shown in Figure 1, where Input is the Input layer, the convolution layer Layer1 is obtained after the convolution operation, and the pooling operation of layer1 is obtained to obtain the pooling layer Layer2, and then the convolution layer of Layer3 and the pooling layer of Layer4 are obtained through the rolling and pooling operations. The final output is classified by the full connection layer.

The typical structure of the convolutional neural network is shown in Figure 4, where Input is the input layer, and the convolutional layer Layer1 is obtained after the convolution operation Layer1 performs the pooling operation to obtain the pooling layer Layer2, and then obtains the convolution layer of Layer3 and the pooling layer of Layer4 through the convolution and pooling operation. Finally, the classification output is carried out by the full connection layer.

### 3.2. Principles of Convolution Pooling

In the convolution stage, the input data are firstly checked through multiple convolution operations, and then a convolution layer composed of multiple feature maps are formed.  Figure 5 shows the convolution process. Assuming that the input data are the two-dimensional array of *i*_1_ × *i*_2_, the input feature map is convolved with n convolution of *k*_1_ × *k*_2_, and then the feature map composed of *N* two-dimensional arrays is output.where *w*_*ij*_ is the weight of each convolution kernel; *y*_*j*_ is the *j*th characteristic graph of the output; *x*_*i*_ is the *i*th feature graph of the input; *J b* is trainable bias; and *F* is the excitation function. The commonly used ReLU excitation function is expressed as follows:

(1) $$\begin{array}{c} \begin{array}{c} y_{j}=f\left(\sum_{i}w_{ij}*x_{i}+b_{i}\right) \end{array}, \end{array}$$

(2) $$\begin{array}{c} f\left(x\right)=\max\left(0,x\right). \end{array}$$

The pooling stage can reduce the dimension of the feature map after convolution, effectively prevent overfitting, and reduce the training parameters, so as to reduce the training time of the model. The commonly used pooling method is max-pooling, whose process principle is shown in Figure 3. In a 4 × 4 feature map, a 2 × 2 filter is used to traverse the feature map with a step size of 2. The maximum value is taken to replace the region traversed by each filter. After traversing, a new 2 × 2 feature map is obtained as shown in the figure.

### 3.3. Logistic Regression

Logistic regression is a common and efficient classifier, which has many advantages, such as no need to assume data distribution in advance and good mathematical properties of the model. The last layer of convolutional neural network is generally the classification layer, and the CNNMDA adopts logistic regression as the classification layer of CNN. The hypothetical function of the logistic regression model is as follows:

(3) $$\begin{array}{c} h_{\theta }\left(x\right)=\frac{1}{1+e^{\theta_{x}^{T}}}. \end{array}$$

This function, also known as the logarithm function, is a differentiable convex function of any order. *h*_*θ*_(*x*) represents the probability of an event for sample *X*, and *θ* is a trainable parameter.

In the dichotomy problem, for a given sample *X*, the probability of belonging to class 0 is as follows:

(4) $$\begin{array}{c} P\left(y=0|x;\theta \right)=1-h_{\theta }\left(x\right). \end{array}$$

The probability of being in class 1 is as follows:

(5) $$\begin{array}{c} P\left(y=0|x;\theta \right)=h_{\theta }\left(x\right). \end{array}$$

For multiclassification problems, the one-VS-all method can be used to transform them into the binary problems.

### 3.4. CNNMDA Data Fusion Algorithm

The CNNMDA algorithm is based on a deep learning model, and the CNN network structure used consists of three convolution layers, one pooling layer, and two full connection layers. Before using the feature extraction model CNNM to fuse node data, the training of the model needs to be completed. The traditional training method is mainly a back propagation algorithm, but the CNNM model needs to modify the back propagation algorithm due to the existence of a convolution layer and pooling layer.

(6) $$\begin{array}{c} \begin{array}{c} J\left(\theta \right)=-\frac{1}{m}\sum_{i=1}^{m}y^{\left(i\right)}\text{In}h_{\theta }\left(x^{\left(i\right)}\right)+\left(1-y^{\left(i\right)}\right)\text{In}\left(1-h_{\theta }\left(x^{\left(i\right)}\right)\right) \end{array}. \end{array}$$

The loss function of CNNM training is

(7) $$\begin{array}{c} \theta_{i}=\theta_{i}-\alpha \frac{\partial }{\partial \theta }J\left(\theta \right). \end{array}$$

The parameters are updated iteratively to minimize the loss function *J*(*θ*), where *θ* is the trainable parameter (including the weight and bias of the convolution kernel), and *α* is the learning rate.

In order to obtain the partial derivative *∂*/*∂θJ*(*θ*) for the convolution layer:

(8) $$\begin{array}{c} \delta_{j}^{l}=\beta_{j}^{l+1}\left(f^{\prime }\left(u_{j}^{l}\right)\cdot \text{up}\left(\delta_{j}^{l}\right)\right), \end{array}$$

where *δ*_*j*_^*l*^ is the sensitivity of the *j*th feature graph of the LTH layer;  *β*_*j*_^*l*+1^ is the parameter of the *j*th feature map of layer *L* + 1. By substituting *δ*_*j*_^*l*^ into equations (8) and (9), the derivative of convolution kernel weight *w* and bias *b* can be obtained.

(9) $$\begin{array}{c} \frac{\partial J}{\partial w_{ij}}=\sum_{uv}{\left(\delta_{j}^{l}\right)}_{uv}{\left(p_{i}^{l-1}\right)}_{uv}, \end{array}$$

(10) $$\begin{array}{c} , \end{array}$$

where (*p*_*i*_^*l*−1^)_*uv*_ is the result of the roll-product operation between the feature map of layer *L* − 1 and the convolutional kernel of layer *L*. At this point, equations (8) and (9) can be substituted into equation (6) to complete a parameter update of the convolution layer.

For the pool layer, there is:

(11) $$\begin{array}{c} z_{j}^{l}=f\left(\beta_{j}^{l}\text{ down }\left(z_{j}^{l-1}\right)+b_{j}^{l}\right), \end{array}$$

(12) $$\begin{array}{c} \delta_{j}^{l}=f\left(\sum_{j=1}^{M}\beta_{j}^{\left(l+1\right)}*k_{ij}\right), \end{array}$$

where *z*_*j*_^*l*^ represents the *j*th feature graph of the *i*th layer; down: performs a pooling operation. The derivative of the weight and bias of the convolution kernel was obtained through equations (10) and (11), as shown in equations (12) and, then the result was substituted into equation (6) to complete a parameter update of the pooling layer.

For the final full connection layer of the convolutional neural network, the traditional back propagation algorithm is still used for training. Formulas (6) are used to improve the backward propagation algorithm, and the training of the CNNM model is completed in combination with the forward propagation process. Finally, the model parameters are obtained, and the CNNMDA can be realized according to the algorithm. The specific algorithm steps are as follows:

1. The sink node extracts the data containing label information from the corresponding database according to the data type to be processed;
2. Input the training data into the constructed CNNM model to begin the training of CNNM, and then the sink node sends the trained parameters to each terminal node through the hair tuft;
3. Each terminal node uses the pretrained CNNM model to carry out multilayer convolution feature extraction and pooling for the collected sensor data, and then send the fusion feature data to the corresponding cluster-head node, in which the process of convolution and pooling is the process of data fusion;
4. The cluster-head node uses logistic regression classifier to classify the fusion data generated in the step (3), get the classification result, and send the fusion data to the sink node;
5. After the network completes a round of data collection, fusion, and transmission, the sink node is reclustered and the cluster-head node is selected, and then jump to the step (3).

Using this algorithm to fuse incoming data of cluster nodes can reduce the amount of outgoing data, thus greatly reducing energy consumption and improving network performance.

## 4. Simulation Experiment

The TensorFlow platform was used to carry out a simulation analysis of the data fusion algorithm. The facility agriculture monitoring system was taken as the application scenario, and the simulation test of the CNNMDA algorithm was completed according to the algorithm in Section 2. In order to highlight the performance of data fusion of the CNNM deep layer model, BPNDA [7], and SOFMDA [8], representative algorithms based on the shallow network model, were used for comparative analysis.

In this section, the ResNet-18 [7] deep neural network model [8] will be used on the Tianhe-2 supercomputer to train the CIFAR-10 data set, bury the runtime steps, and record the key data. The validity of the algorithm is verified by comparing the dynamic data allocation algorithm under the condition of multimachine synchronization and parallelism.

The simulation parameters are shown in Table 2, where the number of nodes and the network range refer to the random distribution of 100 sensor nodes in the perception region of 100, m × 100, and *m* [7].In order to compare the efficiency of each data fusion algorithm, the unoptimized LEACH [15] protocol is adopted, and the energy consumption of data transmission, receiving, and fusion of nodes is counted according to the first kind of wireless communication energy consumption model [16].

The error rate of feature extraction and classification of each algorithm is shown in Table 2, where n, D, and C, respectively, represent the number of network layers of the BP network model, the dimension of input data, and the number of data classification. As can be seen from Table 2, for low-dimensional data with few categories, the error rate of feature extraction and classification of the CNNMDA algorithm is basically the same as that of BPNDA and SOFMDA. With the increase of the input data dimension, the number of parameters of the shallow model BP and SOFM increases sharply, and the performance begins to decline, leading to a significant increase in the error rate. In contrast, the error rate of CNNMDA based on the depth model is always kept at a low level.

### 4.1. Introduction to the Experimental Platform

Tianhe-2 supercomputer has been led by the National University of Defense Technology together with other scientific research units of the heterogeneous supercomputer since June 2013 at a peak speed of 549 million times per second. Continuous computing speed of 339 million times per second double-precision floating point arithmetic is superior performance to become the world's fastest supercomputer and won the top 500 list of global supercomputers six consecutive times. In this experiment, the CPU partition of the high performance computing service of Tianhe-2 is used. This partition has a total of 17920 compute nodes, and each node is equipped with two Intel Xeon E5-2692V2 12-core CENTRAL processing units (CPUs) with the main frequency of 2.2 GHz. The peak performance of the single-CPU double-precision floating point can reach 211.2 GF, and the peak performance of the calculating node can reach 3.432 TF. The memory capacity of each node is 64 GB, the total memory capacity is 1.4 PB, and the external storage is a 12.4 PB hard disk array. The nodes are connected via PCI-E2.0 built into Intel's IvyBridge microarchitecture with a single channel bandwidth of 10GB/ps, providing strong support for cross-node data communication.

MXNet requires gliBC version 2.17 by default. The environment of Tianhe-2 supercomputer does not meet this requirement. Therefore, this experiment needs to recompile MXNet and configure openBLas, LAPACK, OpencV and other environments before editing and translating. This test needs to be carried out in a distributed way. When compiling and translating, set USE_DIST_KVSTORE = 1, and USE SSH to start and stop the server, worker, and scheduler on each computing node.

### 4.2. Experimental Settings

All the deep neural network models used were ResNet-18, the data set used was CIFAR -10, the learning rate was set to 0.1, the optimizer used was SGD, and the momentum was set to 0.9. In this experiment, the main measurement indicators are as follows: (1) Single iteration time (SingleEpochTimeCost): it indicates the total time of the model training in a single epoch. (2) Accuracy: it refers to the prediction Accuracy of a single model for a batch sample of a test set using the current training model after a certain number of iterations during the training process. (3) Total training time (TrainingTimeCost): it represents the number of iterations of the same model and the total length of training time of the model.

### 4.3. CNNMDA Result Analysis

By using EEMD decomposition to decompose the Sse index, 14 IMF components and 1 residual component can be obtained. The IMFl∼IMFl4 correlation coefficient measures the correlation degree between the EEMD decomposed components and the upper index. The correlation coefficients between the IMFl∼IMF4 components and the SSE index are all less than O.1, while the correlation coefficients between IMF5∼IMF9 components and the SSE Index are all in O.1 component and the residual component RES, respectively, showing the fluctuation characteristics of the SSE Index at different time scales from high frequency to low frequency, as shown in Figure 6. As can be seen from Figure 7, the fluctuation frequency from the IMFl component to the IMFl4 component gradually decreases. Among them, the IMFl∼IMF6 component has a higher frequency rate, a smaller amplitude, and a relatively large fluctuation degree, which reflects the drastic fluctuation and fluctuation details of the upper index in a short period. The frequency of IMF7∼IMFl4 components is low, the amplitude is large, and the fluctuation degree is relatively small, which reflects the changing trend of the Shanghai Composite Index in the medium and long term, but the details of the fluctuation of the index are less described. The residual RES component reflects the overall change trend of the Shanghai Composite Index in the long term. Furthermore, the relationship between the IMF component, the RES residual term, and the SSE index is given from the three dimensions of the correlation coefficient, variance contribution rate, and run number in Figures 7(a) and 7.

### 4.4. Comparative Experimental Analysis

#### 4.4.1. Average backward time

Because the WASP protocol adopts weighted gradient and forced synchronization operations, it is inevitable to incur additional time cost during training.  Figure 8 shows the average backward time obtained using different training protocols. For the LENet-5 model using the MINST data set, the average backward time of WASP is much lower than that of BSP and N-soft, but slightly higher than that of ASP. When the number of workers is small (1 4), compared with the ASP, the time cost increase is not significant. When the number of workers is relatively large (entry = 16), the average backward time increases by 0.018 s, which is a relatively small increase.

For the ResNet-101 model using the CIFAR-10 data set, the gradient calculation accounted for a larger proportion of the backward time. Therefore, the weighted operation added by WASP during the gradient application phase has little effect on the backward time. As shown in Figure 9, the time gap between these four training protocols is small. The WASP protocol is only O.175 s longer than the ASP protocol; that is, the time cost increases O.02%.

#### 4.4.2. Training error rate

We use the number of iterations as the cross marker, and the time of each iteration varies according to the protocol. As a representative result of the lenet-5 model, Figure 9 shows the training error rate obtained for different training protocols at the time of entering I-16. We can observe that the training error rate for WASP drops faster at the beginning than for the other protocols. When the number of iterations is about 1 500, the training error rate of WASP gradually approaches O, which is much lower than other training protocols. Although WASP's convergence fluctuates slightly, it is more stable than ASP. With a limited number of iterations, WASP can finally achieve the same convergence as the BSP protocol.

## 5. Conclusions

In this paper, the deep learning model is applied in the field of WSN data fusion, and the data fusion algorithm CNNMDA with the convolutional neural network model as the core is proposed. Simulation experiments show that compared with the traditional fusion algorithms based on BP, SOFM, and other shallow network models, the CNNMDA takes the CNN structure in the deep layer model as the feature extraction model, which can effectively improve the data acquisition accuracy, reduce the error rate, greatly reduce the network communication data and node energy consumption, and prolong the network life cycle by which a good fusion effect was obtained. The Deep learning model has a broad application prospect in the field of data fusion. How to better simplify model parameters and improve algorithm execution efficiency still needs more in-depth research.

After using the dynamic data allocation algorithm under multimachine synchronization and parallel, the training speed of the CNNMDA model has been significantly improved, and it can approach the accuracy of synchronous mode. Compared with the traditional synchronization mode, the main advantage of the proposed algorithm is that it improves the training speed. Its essence is to reduce the waiting time of nodes with high performance and eliminate the shortboard effect brought by the synchronization mode. Compared with the traditional asynchronous mode, the convergence of the model is better guaranteed. Therefore, the dynamic data allocation algorithm in this paper achieves the expected results under multimachine synchronization and parallel.

## Figures and Tables

**Figure 1:** The processing flow of computing nodes.

**Figure 2:** Flow chart of the data of the software.

**Figure 3:** The processing flow of parameter server nodes.

**Figure 4:** Structure of convolutional neural network.

**Figure 5:** Workflow of convolution phase.

**Figure 6:** Decomposition of CNNMDA.

**Figure 7:** Accuracy comparison of the CNNMDA (a). Loss comparison diagram (b).

**Figure 8:** Average backward time of the CNNMDA.

**Figure 9:** Training error of the CNNMDA.

**Table 1:** Meaning of related parameters in the algorithm.

Parameters	Describe

start_*i*_	The starting point for data assignment on compute node *i*
end_**i**_	The termination point of data assignment on compute node *i*
len	The total number of samples
*i*	The *i*th compute node
batchsize_**i**_	Batch size of compute node *i*
speed_**i**_	The training speed of node *i*

**Table 2:** Simulation parameters.

Parameters	Value

Network range	100 × 100
Number of nodes	100
Coordinate of sink node	50, 50
Node initial energy	0.5
Convolution kernel size	3 × 3
Packet length	2000
The length of the cluster message	100
The length of the Baotou	100
Maximum number of simulation wheels	2000
Convolution step	1

## Data Availability

The data used to support the findings of this study are available from the corresponding author upon request.
